This article has been retracted.

# Health and Nutrition Literacy and Adherence to Treatment in Children, Adolescents, and Young Adults With Chronic Kidney Disease and Hypertension, North Carolina, 2015

**DOI:** 10.5888/pcd13.160044

**Published:** 2016-08-04

**Authors:** Nikita Patel, Maria Ferris, Eniko Rak

**Affiliations:** Author Affiliations: Maria Ferris, Eniko Rak, The University of North Carolina at Chapel Hill School of Medicine, Chapel Hill, North Carolina.

## Abstract

**Introduction:**

Adherence to treatment and dietary restrictions is important for health outcomes of patients with chronic/end-stage kidney disease and hypertension. The relationship of adherence with nutritional and health literacy in children, adolescents, and young adults is not well understood. The current study examined the relationship of health literacy, nutrition knowledge, nutrition knowledge–behavior concordance, and medication adherence in a sample of children and young people with chronic/end-stage kidney disease and hypertension.

**Methods:**

We enrolled 74 patients (aged 7–29 y) with a diagnosis of chronic/end-stage kidney disease and hypertension from the University of North Carolina Kidney Center. Participants completed instruments of nutrition literacy (Disease-Specific Nutrition Knowledge Test), health literacy (Newest Vital Sign), nutrition behavior (Nutrition Knowledge–Behavior Concordance Scale), and medication adherence (Morisky Medication Adherence Scale). Linear and binary logistic regressions were used to test the associations.

**Results:**

In univariate comparisons, nutrition knowledge was significantly higher in people with adequate health literacy. Medication adherence was related to nutrition knowledge and nutrition knowledge–behavior concordance. Multivariate regression models demonstrated that knowledge of disease-specific nutrition restrictions did not significantly predict nutrition knowledge–behavior concordance scores. In logistic regression, knowledge of nutrition restrictions did not significantly predict medication adherence. Lastly, health literacy and nutrition knowledge–behavior concordance were significant predictors of medication adherence.

**Conclusion:**

Nutrition knowledge and health literacy skills are positively associated. Nutrition knowledge, health literacy, and nutrition knowledge–behavior concordance are positively related to medication adherence. Future research should focus on additional factors that may predict disease-specific nutrition behavior (adherence to dietary restrictions) in children and young people with chronic conditions.

## Introduction

Chronic kidney disease/end-stage kidney disease (CKD/ESKD) and hypertension require adherence to a complicated medication regimen (1) and dietary restrictions. Low-sodium foods, to reduce blood pressure and volume overload, are prescribed with both conditions. With CKD/ESKD, phosphorus intake should also be reduced (2) to maintain growth and prevent cardiovascular complications (3). Yet, for many, adherence to treatment is a significant challenge (4).

Health literacy is one of the most influential factors of treatment adherence in young patients with chronic conditions (5). Health literacy is the ability of individuals to obtain, process, and understand basic health information and services to make informed health decisions (6,7). Health literacy has been explored in relation to various health outcomes in adolescents and young adults (8), but research is lacking on its impact on nutritional behavior and adherence to dietary regimens in children, adolescents, and young adults with chronic conditions (9). At least 1 in 3 adolescents have low health literacy (5), compromising their ability to process information provided on prescription and nutrition labels (10).

The objective of this study was to examine the relationship of health literacy, disease-specific nutrition literacy, nutrition knowledge–behavior concordance (KBC) and treatment adherence in children, adolescents, and young adults seen at the UNC Kidney Center. We hypothesized that 1) young individuals with adequate health literacy will have better disease-specific nutrition knowledge and higher nutrition KBC scores; 2) young individuals with higher medication adherence scores will have better disease-specific nutrition knowledge and nutrition KBC; 3) young individuals with better health literacy will have higher adherence scores; 4) health literacy and nutrition knowledge can significantly predict nutrition KBC and 5) health literacy, nutrition knowledge, and nutrition KBC are significant predictors of medication adherence.

## Methods

Patients treated at the pediatric and adult clinics of the UNC Kidney Center (a Southeastern US nephrology practice) participated in this study approved by the University of North Carolina institutional review board. A sample of 74 patients aged 7 to 29 years with hypertension or CKD/ESKD (stages 1 to 5, including transplant) were enrolled from May 2015 through September 2015. This age group was chosen because habits and behaviors are still forming, making this age range an important period for lifelong health-related behaviors and attitudes (11). CKD stage was determined by the patient’s estimated glomerular filtration rate (eGFR) based on the Schwartz equation for children (12). The clinic’s registry was used to identify potential participants. Participants were approached at the time of the clinic visit and invited to participate. Consents, assents, and parental permission were obtained in person at the time of enrollment. Trained research assistants collected all data during in-person interviews.

Participants were administered the Newest Vital Sign (13), a 6-item tool that measures literacy and numeracy skills through interpretations of an ice cream food label. Patients answer 6 questions based on information presented on the label. The instrument has been validated in patients over the age of 7 (14) and is used in studies to measure health literacy in children (11). Scores ranging from 0 to 6 were transformed into a categorical measure, yielding 3 literacy levels: high likelihood of limited literacy (score of 0 or 1), possibility of limited literacy (score of 2 or 3), and adequate literacy (score of 4, 5, or 6). For our research, we collapsed the inadequate literacy groups (scores of 0–3) into a single category, because few participants scored in the lowest category, creating 2 groups: youths with inadequate health literacy levels and youths with adequate health literacy levels. This measure was administered verbally to patients.

The Morisky Medication Adherence Scale (MMAS-8) (15) was used to evaluate medication adherence. The MMAS-8 is an 8-item questionnaire that is accessible for use in clinical settings to monitor adherence and to identify patients with adherence problems. A score of 0 indicates a high level of adherence, a score of 1 or 2 indicates moderate adherence, and a score of 3 to 8 indicates low adherence. This measure was administered verbally to the patients. In our analysis, we created a dichotomous variable that differentiated between those who were adherent (score of 0 on the scale) and those who were nonadherent (a score of 1 or above).

The disease-specific knowledge questionnaire was adapted from our CKD Knowledge Test developed in-house (16) at Ferris Laboratory as part of the pilot assessment of the CKD Knowledge and Self-Management web-based game called Planet K, a telephone application for an ongoing interventional trial funded by the Centers for Disease Control and Prevention. Seven questions were used to assess patients’ understanding of the dietary restrictions relating to their own diagnosis (hypertension or chronic kidney disease). The number of correct responses was summed, yielding a continuous variable, ranging from 0 to 7.

The Disease-Specific Nutrition-Knowledge Behavior Concordance activity was created for this study to determine the concordance of nutrition/dietary knowledge with nutrition behavior on the basis of recommendations for hypertension and chronic kidney disease diets from the National Kidney Foundation (2). Ten pairs of pictures were shown to the patient, with one picture in each pair being the healthy food item and the other depicting the unhealthy food item respective to their condition. We showed participants the pairs to measure their eating habits as well as their dietary knowledge. We tested their food consumption behaviors before testing their nutrition knowledge, using the same pair of pictures, to reduce social desirability response bias. Participants were asked to pick the food item (from each pair) that they ate more commonly (measuring behavior). A healthier choice yielded a correct response to the items, or a score of 1 point. Correct responses were summed. Scores on the behavior scale ranged from 0 to 10. Next we tested knowledge of dietary restrictions. The same picture-pairs were shown again, and participants were prompted to select the food item that they should avoid to stay healthy when living with hypertension or chronic kidney disease. For example, we showed a picture of chicken nuggets with ketchup next to a picture of grilled chicken. The knowledge question asked, “Which one is a better option as a meal?” and the behavior question asked, “Which one are you more likely to eat?”

To compute the concordance score, we combined the knowledge and behavior scores. A value of 1 was assigned to No Correct Knowledge and No Desirable Food Consumption Behavior; a 2 was given for Correct Knowledge and No Desirable Behavior; a 3 for No Correct Knowledge and Desirable Behavior, and a 4 for Correct Knowledge and Positive Behavior. On the 10 pairs, participants may have scored a value of 1 to 4 depending on the combination of their nutrition knowledge and behavior score. We summed the scores across the 10 concordance items to compute the nutrition knowledge–behavior concordance variable that ranged from 10 to 40. Higher scores meant that patients knew what they should eat and demonstrated healthy dietary habits as well. Low scores meant no knowledge and poor eating habits.

### Data analyses

To test hypothesis 1, we performed univariate tests, including χ^2^ and independent sample *t* tests to compare scores on nutrition knowledge and nutrition knowledge–behavior concordance of those with inadequate and adequate health literacy skills. We used the same methodology for the second hypothesis, with adherence as our grouping variable. For our third hypothesis, χ^2^ analysis was used to understand how health literacy relates to adherence (both measures dichotomous). For hypothesis 4, we employed multivariate linear and binary logistic regression tests to determine if health literacy and disease-specific nutrition knowledge predict nutrition knowledge–behavior concordance and medication adherence, controlling for age, race, sex, and type of insurance. We also tested behavior only (from the nutrition knowledge–behavior concordance composite). For hypothesis 5, logistic regression tested whether health literacy and nutrition knowledge predict adherence (as a dichotomous outcome), and linear regression examined if these predictors contribute to explaining nutrition knowledge–behavior concordance (as a continuous measure), again controlling for age, race, sex, and type of insurance. Significance was determined at *P* < .05 for all analyses. SPSS Statistics 22 (IBM Corp.) was used to analyze the data.

## Results

### Participant characteristics

We enrolled 74 patients, which included children, adolescents, and young adults with a mean age of 18.5 (standard deviation [SD], 6 y) (Table 1). Children, defined as aged 18 years or younger, constituted 51.4% of the sample (n = 38), and adults, defined as aged 18 or older, constituted 48.6% of the sample (n = 36). Females (58.1%) represented the majority of the sample. White (44.6%) was the most common race/ethnicity, followed by African American (29.7%), and other race/ethnicity (25.7%). Half of the sample had private insurance (50.0%), 31.9% had public insurance, 15.3% had both private and public insurance, and 2.8% had no insurance. Of the participants enrolled, 58.1% had chronic kidney disease and 41.9% had hypertension. 

**Table 1:** Population Characteristics of Children, Adolescents, and Young Adults With Chronic Kidney Disease and Hypertension (n = 74), North Carolina, 2015^a^

Characteristic	No. (%)
**Mean age (SD), y**	18.5 (6)
**Age group**	
Children (aged <18 y)	38 (51.4)
Adult (aged ≥18 y)	36 (48.6)
**Sex**	
Male	31 (41.9)
Female	43 (58.1)
**Diagnosis**	
Chronic kidney disease stages 1–5^b^	43 (58.1)
Stage 1	7 (16.3)
Stage 2	6 (14.0)
Stage 3	11 (25.6)
Stage 4	3 (20.9)
Stage 5	16 (37.2)
Hypertension	31 (41.9)
**Race/ethnicity**	
White	33 (44.6)
African American	22 (29.7)
Other (Hispanic, Asian, mixed, other)	19 (25.7)
**Insurance^c^**	
Private	36 (50.0)
Public	23 (31.9)
Both (private and public)	11 (15.3)
No insurance	2 (2.8)
**Individualized education plan (IEP) status^d^**	
IEP	13 (41.9)
No IEP	18 (58.1)

Abbreviation: SD, standard deviation.

a All values are number (percentage) unless otherwise indicated.

b Chronic kidney disease subdivided by stage.

c Data missing for 2 participants.

d Only children in grade school had individualized education plans. Not all participants in the study provided a response.

An examination of associations between demographic variables and variables of interest for the study (health and nutrition literacy, nutrition knowledge, nutrition knowledge–behavior concordance, and adherence) revealed some important differences. Age was found to have an important role in developing these competencies. A higher proportion of adults scored adequately on the health literacy measure (χ^2^ = 6.5, *P* = .01). In addition, the averages of disease-specific nutrition knowledge scores of adults were significantly higher than for children/adolescents (mean, 5.6 [SD, 1.2]) vs (mean, 4.4 [SD, 1.3]), and the results on the disease-specific nutrition knowledge–behavior concordance scores were similar for children (mean, 29.6 [SD, 3.9]) and adults (mean, 31.5 [SD, 4.0]). More patients with private insurance scored adequate on health literacy (χ^2^ = 10.9, *P* = .001) than their counterparts with public, mixed, or no insurance. The mean nutrition knowledge scores and the nutrition knowledge–behavior concordance scores of patients in the private insurance category was similar to those of patients in the public/no insurance group. We found slightly higher proportions of white participants in the adequate literacy group (χ^2^ = 3.6, *P* = .06). Sex was not associated with literacy or nutrition knowledge scores in this sample.

### Differences in nutrition knowledge and nutrition knowledge–behavior concordance scores

For our first hypothesis, nutrition knowledge scores were significantly higher for participants with adequate health literacy compared with participants with inadequate literacy (*P* = .01) (Table 2). However, health literacy did not significantly affect nutritional knowledge–behavior concordance (*P* = .40). For our second hypothesis, nutrition knowledge scores (*P* = .04) and nutrition knowledge–behavior concordance scores (*P* = .001) varied significantly between groups, and greater adherence was significantly associated with higher average scores on the nutrition knowledge and knowledge–behavior measures. For our third hypothesis, χ^2^ test results indicated that those with higher health literacy have significantly greater medication adherence (χ^2^ = 7.7, *P* = .006).

**Table 2:** Differences in Nutrition Knowledge and Nutrition Knowledge–Behavior Concordance (KBC) by Literacy Level and Medication Adherence^a^

Measure	Difference	*t* (*df*)	*P* Value	Mean Score (SD)	Mean Score (SD)
**Literacy level**				**Inadequate literacy (n = 36)**	**Adequate literacy (n = 38)**
Nutrition knowledge	−0.81	−2.54 (72)	.01	4.6 (1.5)	5.4 (1.3)
Nutrition KBC	−0.81	−0.85 (72)	.40	30.1 (4.2)	30.9 (3.9)
**Medication adherence**				**Nonadherent (n = 40)**	**Adherent (n = 30)**
Nutrition knowledge^b^	−0.71	−2.09 (68)	.04	4.7 (1.4)	5.4 (1.4)
Nutrition KBC^c^	−3.03	−3.32 (68)	.001	29.3 (4.1)	32.3 (3.3)

Abbreviation: *df*, degrees of freedom.

a Ns vary because data were missing for some study participants.

b Knowledge score based on disease-specific nutrition questionnaire (scores range from 0 to 7).

c Knowledge–behavior concordance (KBC) scores based on a composite of knowledge and behavior scores in a disease-specific nutrition activity (scores range from 10 to 40).

Health literacy was not included in the model for our fourth hypothesis because the univariate associations were not significant. In the multivariate model, nutrition knowledge was not a significant predictor of nutrition behavior (β = 0.09; *P* = .47) or nutrition knowledge–behavior concordance (β = 0.12; *P* = .33).

The results of logistic regression (Table 3), examining the role of health literacy and nutrition knowledge-behavior concordance in predicting adherence (the fifth hypothesis), showed that health literacy is a significant predictor of medication adherence. Nutrition knowledge was not a significant predictor, but the nutrition knowledge–behavior concordance score was a significant predictor of adherence. The odds of adherence increased significantly for those with adequate health literacy, and we also found better medication adherence in those with higher nutrition knowledge-behavior concordance.

**Table 3:** Logistic Regression Testing Health Literacy and Nutrition Knowledge as Predictors of Medication Adherence

Predictor	OR (95% CI)	*P* Value
**Nutrition knowledge as predictor of medication adherence**		
Sex (female)^a^	0.67 (0.22–2.06)	.49
Race (other)^b^	0.77 (0.22–2.70)	.61
Age	1.29 (0.65–2.55)	.48
Insurance (public or none)^c^	3.24 (0.77–13.63)	.09
Nutrition knowledge	1.22 (0.79–1.88)	.33
Health literacy (adequate)^d^	4.97^e^ (1.28–19.34)	.02^e^
Model fit χ^2^_7_ = 3.6, *P* =.83		
**Nutrition knowledge-behavior as predictor of medication adherence**		
Sex (female)^a^	0.54 (0.16–1.80)	.37
Race (other)^b^	0.74 (0.20–2.71)	.59
Age	1.19 (0.74–1.91)	.91
Insurance (public or none)^c^	3.76 (0.79–17.79)	.06
Nutrition knowledge–behavior concordance	1.29 (1.09–1.53)	<.001^e^
Health literacy (adequate)^d^	6.49 (1.45–28.98)	.01^e^

a Referent group is male.

b Referent group is white.

c Referent group is private insurance.

d Referent group is low health literacy.

e Goodness-of-fit was tested with Hosmer and Lemeshow test. Model fit χ^2^_8_ = 5.0, *P* = .76.

## Discussion

Our study found that health literacy (based on interpretations of a food label) in this cohort of youths with CKD/ESKD or hypertension was related to their understanding of disease-specific dietary restrictions. Inadequate health literacy skills, reflected in the inability to interpret a food label (Newest Vital Sign), were associated with more limited understanding of disease-specific dietary restrictions. Inadequate health literacy skills affect health outcomes in various ways (5). Inadequate health literacy skills provide a barrier to understanding nutrition and could limit a young patient’s understanding of healthy food practices in the context of their disease. A study of health literacy and medication adherence in kidney transplant recipients found that better health literacy improves patients’ medication adherence or transplant outcomes (17). This finding, along with the findings that health literacy predicts disease-specific nutrition knowledge, suggests that poor health literacy could be a barrier for young patients in managing their disease. Specifically, the inability to interpret a food label can limit patients’ ability to understand what they should and should not consume, which in turn affects their ability to adhere to dietary regimes as prescribed by health care professionals (18). Adolescents with poor health literacy have higher odds of obesity, suggesting a link between health literacy and chronic disease (19). This study highlights some benefits of assessing patients’ health literacy. Health professionals should evaluate the literacy level of chronically ill young patients and adjust service delivery approaches, including patient education, accordingly.

As expected, this study found that patients with better medication adherence also had better disease-specific nutrition management (nutrition knowledge–behavior concordance scores); they had higher scores on dietary restriction knowledge as well as food consumption behavior. This finding suggests that patients who feel more able to manage their medication are more likely to focus on every aspect of their disease management, including adhering to dietary restrictions and healthy nutritional practices. Medication-adherent patients were more health-literate and showed higher nutrition knowledge–behavior concordance.

Interestingly, nutrition behavior did not differ between those with adequate health literacy and those with inadequate health literacy. We hypothesized that patients with better understanding of their disease-specific dietary restrictions would have healthier eating habits. However, we found that knowledge did not significantly predict nutritional knowledge–behavior concordance. Similar findings have been found in adults (20), suggesting that other factors could be influential for adopting and maintaining healthy nutritional behaviors and should be considered in young adults who have chronic health conditions. Nutrition education alone does not necessarily improve dietary compliance. Studies of dietary adherence in adults with chronic kidney disease have found that socioeconomic status, knowledge of renal diet, attitudes toward the renal diet and its effectiveness, and proper education are factors that influence adherence (21). With children, the complexity increases with variables including lack of family support, low level of education, cultural and socioeconomic variability, rebellion against strong parental supervision, and denial of disease diagnosis (22). Youssef et al (23) found that a nutrition education intervention significantly improved nutrition knowledge among children on regular hemodialysis, but attitudes and eating habits or practices did not change. Knowledge of proper nutritional practice, along with young adults’ self-efficacy, including disease-management self-efficacy, motivation for change, and family environment, can also be considered in determining how well young patients would follow their dietary restrictions (9). Although many variables were tested in this study (demographic, literacy, disease-specific diet knowledge), future research should focus on additional factors that can fully explain nutritional behavior and dietary restriction adherence.

Our study had limitations. We conducted our study in a single center, in 2 different practices, limiting the generalizability of our study. However, the sample was well distributed by race/ethnicity, insurance type, and sex. Future studies with a larger sample from different centers and more geographically diverse locations are needed. Another limitation of our study was the broad age range of our population. Future studies should stratify samples by age (eg, children, young adults) to determine implications for each age group. The answers to the questionnaires for medication adherence and behavior were self-reported, which inherently has bias.

Our study highlights the need for nutrition-based instruction for patients with chronic conditions that accounts for literacy level. In addition to exploring factors affecting nutritional behavior, future studies should also include designing programs or interventions to effectively guide providers when counseling their patient to focus on nutrition education. Future studies should focus on finding barriers to patients’ understanding and implementing adherence to dietary restrictions. Future analysis should also assess caregivers’ involvement and how caregivers’ food practices could explain the food behavior of young patients.
